The article "Identification of Clinical Prognostic Regulators and Analysis of Ferroptosis-Related Signatures in the Tumor Immune Microenvironment in Lung Squamous Cell Carcinoma" was retracted in 2023. Reasons: unreliable results or conclusions; lack of ethics approval or compliance; concerns about the data; concerns about the peer review.

# Identification of Clinical Prognostic Regulators and Analysis of Ferroptosis-Related Signatures in the Tumor Immune Microenvironment in Lung Squamous Cell Carcinoma

**DOI:** 10.1155/2023/9155944

**Published:** 2023-02-15

**Authors:** Wentao Wang, Guanghui Cui, Song Zhao

**Affiliations:** Department of Thoracic Surgery, First Affiliated Hospital of Zhengzhou University, No. 1, Longhu Middle Ring Road, Jinshui District, Zhengzhou City, Henan Province, China

## Abstract

**Objective:**

Lung squamous cell carcinoma (LUSC) is a common respiratory malignancy and presents an increasing prevalence. Ferroptosis is a newly identified controlled cell death that has captured clinical attention worldwide. However, the ferroptosis-related lncRNA expression in LUSC and its relevance to prognosis remain elusive.

**Methods:**

The research measured predictive ferroptosis-related lncRNAs in LUSC samples from the TCGA datasets. Data on the stemness indices (mRNAsi) and corresponding clinical characteristics were obtained from TCGA. A prognosis model was established using the LASSO regression. Changes within the neoplasm microenvironment (TME) and medicine association were examined to grasp higher immune cell infiltration in numerous risk teams. In line with coexpression studies, the expression of lncRNAs is closely associated with that of ferroptosis. They were overexpressed in unsound people in the absence of alternative clinical symptoms.

**Results:**

The low-risk and speculative teams were considered to have substantial differences in CCR and inflammation-promoting genes. C10orf55, AC016924.1, AL161431.1, LUCAT1, AC104248.1, and MIR3945HG were highly expressed in the high-risk group, suggesting their involvement in the oncology process of LUSC. Moreover, AP006545.2 and AL122125.1 were considerably higher in the low-risk group, implying the potential of these genes as LUSC tumor suppressor genes. The biomarkers listed above may serve as therapeutic targets for LUSC. lncRNAs were also linked to patient outcomes in the LUSC trial.

**Conclusion:**

lncRNAs of ferroptosis were overexpressed in the high-risk cohort without other clinical signs, implying their potential to predict BLCA prognosis. GSEA highlighted immunological and tumor-related pathways in the high-risk group. LUSC occurrence and progression are linked to lncRNAs of ferroptosis. Corresponding prognostic models help forecast the prognosis of LUSC patients. lncRNAs of ferroptosis and associated immune cell infiltration in the tumor microenvironment (TME) may serve as potential therapeutic targets in LUSC, which requires further trials. In addition, the lncRNAs of ferroptosis signature offer a viable alternative to predict LUSC, and these ferroptosis-lncRNAs show a prospective research area for LUSC-targeted treatment in the future.

The article "Identification of Clinical Prognostic Regulators and Analysis of Ferroptosis-Related Signatures in the Tumor Immune Microenvironment in Lung Squamous Cell Carcinoma" was retracted in 2023. Reasons: unreliable results or conclusions; lack of ethics approval or compliance; concerns about the data; concerns about the peer review.

## 1. Background

Lung cancer is divided into two microscopic anatomy groups that differ clinically [1]. Lung squamous cell carcinoma (LUSC) occupies 40-51% of lung cancer types [2] and is affected by age, sex, and smoking. LUSC features a slow development and is mostly surgically resected in the early stage of disease, resulting in a good 5-year survival of patients [3]. Radiotherapy and chemotherapy are considered more effective for the management of LUSC versus small cell undifferentiated carcinoma. Recent improvements in molecular research and medication advancement have accelerated progress for LUSC management. However, current therapeutic targets are susceptible to resistance [4]. Therefore, there exists a pressing need to identify novel and reliable biomarkers for the early identification and diagnosis of LUSC.

It has been demonstrated that lncRNAs feature multiple biological functions, such as tumorigenesis [5, 6]. Iron-dependent lipid peroxidation promotes ferroptosis. A growing body of data implies that ferroptosis regulatory genes play a role in tumor growth. Furthermore, ferroptosis inducer enhances the efficiency of chemotherapy medicines against a variety of malignancies. Ferroptosis is promoted by glutathione depletion, decreased glutathione peroxidase activity (GPX4), and the inability to conduct glutathione reductase metabolism mediated by GPX4, resulting in the formation of reactive oxygen species from divalent iron oxide lipids and cell death [7, 8]. Ferroptosis is available for various disorders. More iron is required in cancer cell growth compared to normal cells, and an imbalance in iron metabolism may accelerate tumor development [9]. Hence, stimulation of the ferroptosis pathway may reverse the resistance to current chemotherapy medicines [10].

lncRNAs are RNA molecules with a high level of expression selectivity. Several studies have discovered that lncRNAs have a variety of biological roles, including gene control, tumor incidence, development, and even metastasis regulation [5, 6]. The lncRNAs may collaborate to boost c-Myc expression and activate the Wnt pathway, which is important in the development of colorectal cancer [11]. Meanwhile, the lncRNA TUG1 was increased in hepatoblastoma, stimulating the downstream signaling pathway of JAK2/STAT3 and promoting angiogenesis in hepatoblastoma cells [12]. The lncRNA HLA complex group 11 has been shown to diminish the malignancy of non-small-cell lung cancer by reducing the expression levels of carcinogenic microRNA875 [13]. However, transfection with lncRNA short nucleolar RNA host gene eight reduced RASA1 expressions, shielding H9C2 cells against HI/R damage [14]. Nonetheless, the association of lncRNAs with immune cell infiltration in ironophilic cell disease is yet unclear. It has been reported that lncRNAs regulate iron droop and govern ferroptosis and apoptosis, while silencing lncRNAs significantly reduces ferroptosis as well as mitigates inflammation and lipid peroxidation [15, 16].

The article "Identification of Clinical Prognostic Regulators and Analysis of Ferroptosis-Related Signatures in the Tumor Immune Microenvironment in Lung Squamous Cell Carcinoma" was retracted in 2023. Reasons: unreliable results or conclusions; lack of ethics approval or compliance; concerns about the data; concerns about the peer review.

## 2. Materials and Methods

The approaches proposed by Wu et al. [17] were adopted in the present study.

### 2.1. Datasets and FRGs

LUSC gene expression patterns and medical data were collected from The Cancer Genome Atlas (TCGA). The expression patterns of 504 LUSC cases and 49 healthy cases were recruited in the TCGA shared database on September 15, 2022. The strategy is to look at gene expression profiles (cases: lung and TCGA and TCGA-LUSC; files: transcriptome profiling and gene expression quantification and HTSeq-FPKM) and clinical research information (cases: lung and TCGA and TCGA-LUSC; files: clinical and bcr xml). In addition, 382 ferroptosis-related genes (FRGs) were obtained from FerrDb [18] (Table 1).

### 2.2. Annotation of lncRNAs

Transcriptome data and human configuration files were acquired using Perl software (https://www.perl.org/), and the target mRNA and lncRNA gene expression data were extracted. Gene IDs were translated to gene names using data from the Ensembl database (http://asia.ensembl.org/info/data/index.html). R4.1.0 limma package was employed to collect FRG expression data.

### 2.3. Ferroptosis-Related lncRNA Identification

Limma package's correlation test was adopted to analyze the expression of ferroptosis-related lncRNAs after normal sample filtering with *p* < 0.001 and corFilter = 0.4 as screening criteria. Connection of FRG expression with lncRNAs was assessed using the coexpression analysis. FDR < 0.05 and |log2FC| ≥ 1 were employed to assess the expression of ferroptosis-related lncRNAs. First, the functions of FRGs that were differentially expressed and were upregulated and downregulated (DEGs) were examined. With Gene Ontology (GO), DEG-related biological pathways were analyzed. Biological processes (BP), molecular functions (MF), and cellular components (CC) controlled by the differentially expressed ferroptosis-related lncRNAs were evaluated based on Kyoto Encyclopedia of Genes and Genomes (KEGG) data using the R clusterProfiler package.

### 2.4. Prognostic Signature for Ferroptosis-Related lncRNAs

A ferroptosis-related lncRNA signature was generated using LASSO-penalized Cox regression and univariate Cox regression analysis, stratified by risk score (coefficient lncRNA_1_ × expression of lncRNA_1_) + (coefficient lncRNA_2_ × expression of lncRNA_2_) +  ^⋯^ + (coefficient lncRNA_*n*_ × expression lncRNA_*n*_). Assessment of the associated risk score of each LUSC patient was performed. The RNAs were dichotomized into low risk (< median number) and high risk (≥ median number) based on their median scores. LASSO regression identified the low-risk (50%) and high-risk (50%) groups, and the corresponding plots were drawn. The forest diagram and survival curves were created. A comparable receiver operating characteristic (ROC) curve was drawn to test the accuracy of the model in predicting survival. Multivariate and univariate models were used to obtain the hazard ratios and assess the association of clinical factors with the risk prediction model. Risk and clinical correlation analyses were completed. Heatmaps and decision curve analysis (DCA) were constructed to further show our model's accuracy.

The article "Identification of Clinical Prognostic Regulators and Analysis of Ferroptosis-Related Signatures in the Tumor Immune Microenvironment in Lung Squamous Cell Carcinoma" was retracted in 2023. Reasons: unreliable results or conclusions; lack of ethics approval or compliance; concerns about the data; concerns about the peer review.

### 2.5. GSEA and Predictive Nomogram

GSEA was used to explore the disparities in related functions and pathways, and data were imported using Perl. Associated scores and graphs were employed to evaluate the dynamic of the functions and routes to the various risk groups. A nomogram was generated through the combination of the predictive signals to predict the 1-, 2-, and 3-year OS of LUSC patients.

### 2.6. Immunity Analysis and Gene Expression

According to ferroptosis-related lncRNA signatures, the CIBERSORT, ESTIMATE, MCPcounter, single-sample gene set enrichment analysis (ssGSEA), and TIMER algorithms were used to compare cellular components or cellular immune responses across the two groups. A heatmap was used to explore alterations in the immune response, and ssGSEA was used to quantify tumor-infiltrating immune cell subgroups and their immunological function.

## 3. Results

### 3.1. FRG Enrichment Analysis

102 DEGs were identified (35 down- and 67 up-). GO analysis revealed 655 core targets. The MF mainly involved iron ion binding (GO:0005506). CC mainly involves the basal part of the cell (GO:0045178). BP involves neuron death (GO:0070997). KEGG analysis was used to identify the primary signaling pathways, which indicated that lncRNAs were mostly engaged in the HIF-1 signaling pathway (hsa04066), ferroptosis (hsa04216), and microRNAs in cancer (hsa05206) (Figure 1).

### 3.2. Prognostic Signature

Five hundred five ferroptosis-related lncRNAs were discovered. Eight important ferroptosis-related lncRNAs were discovered within the univariate and variable Cox analyses. Overall, eight completely different lncRNAs (C10orf55, AC016924.1, AL161431.1, AP006545.2, LUCAT1, AC104248.1, AL122125.1, and MIR3945HG) were discovered to be freelance LUSC prognostic indicators (Figure 2). As a result, we tended to compute risk ratings and create a prognostic signature.

The article "Identification of Clinical Prognostic Regulators and Analysis of Ferroptosis-Related Signatures in the Tumor Immune Microenvironment in Lung Squamous Cell Carcinoma" was retracted in 2023. Reasons: unreliable results or conclusions; lack of ethics approval or compliance; concerns about the data; concerns about the peer review.

### 3.3. Survival Results

The presence of high-risk lncRNA signatures was related to a lower survival rate (*p* < 0.001, Figure 3(a)). The AUC of signature was 0.658, suggesting a better predictive value for LUSC prognosis than standard clinicopathological variables (Figures 3(b) and 3(c)). Risk scores of the patient were correlated with LUSC patient survival. Surprisingly, most lncRNAs discovered in the present study correlated negatively with the risk model (Figure 3(d)). The AUCs of signature for 1-, 2-, and 3-year survival rates were 0.658, 0.693, and 0.687 (Figure 3(e)). We examined the data and found that most of the patients had a large gap in survival years, which may have contributed to the AUC being less than 0.7. High expression of AC104248.1, C10orf55, LUCAT1, AL161431.1, AC016924.1, and MIR3945HG was found in the high-risk group, implying their negative impacts on the prognosis of LUSC patients (Figure 3(f)). lncRNA signature (HR: 1.434, 95% CI: 1.315-1.565), age (HR: 1.022, 95% CI: 1.005-1.039), and tumor stage (HR: 1.242, 95% CI: 1.050-1.470) were independent risk factors for prognosis (Figures 4(a)–4(c)).  Figure 5 shows the heatmap for the prognosis signature. C10orf55, AC016924.1, AL161431.1, LUCAT1, AC104248.1, and MIR3945HG were found in the high-risk group. AP006545.2 and AL122125.1 were found in the low-risk group. The hybrid nomogram was accurate, which demonstrated great potential in the therapy of LUSC patients (Figure 6).

### 3.4. GSEA

According to GSEA, ferroptosis-related lncRNAs are predictive markers for immunological and tumor-related pathways, such as graft versus host disease, allograft rejection, asthma, type 1 diabetes mellitus, NOD-like receptor signaling pathway, chemokine signaling pathway, and JAK-STAT signaling pathway. The top 6 enriched functions or pathways for each cluster are shown in Figure 7. As a consequence, “NOD-like receptor signaling pathway” was the most enriched, and some of the genes were positively correlated with “H” or “L.”

### 3.5. Immunity and Gene Expression

Figure 8 demonstrates a heatmap of the immunological responses generated. Correlation analysis using ssGSEA showed that the two groups differed significantly in terms of CCR, inflammation-promoting, and other immune cell subpopulations and related activities (Figure 9(a)). It can be seen that there are many kinds of immune cell infiltration in LUSC patients. These may be a target for future therapies. In immune checkpoints, significant discrepancies were identified in the expression of TMIGD2, TNFRSF4, CD244, NRP1, and CD276 (Figure 9(b)). The expression of YTHDF1, METTL3, FTO, HNRNPC, and YTHDC1 was significant between the two groups (Figure 10). These genes should be the focus of future research; they are not only related to iron death but also related to mRNA modification.

The article "Identification of Clinical Prognostic Regulators and Analysis of Ferroptosis-Related Signatures in the Tumor Immune Microenvironment in Lung Squamous Cell Carcinoma" was retracted in 2023. Reasons: unreliable results or conclusions; lack of ethics approval or compliance; concerns about the data; concerns about the peer review.

## 4. Discussion

With the aging of the population, changes in lifestyle, and environmental degradation, the prevalence of LUSC in China has grown year after year, and LUSC treatment is a serious clinical concern [19]. Ferroptosis is associated with abnormal cell death in LUSC. Previous research has linked ferroptosis to aberrant death in chronic disorders, and ferroptosis has also been demonstrated to impart therapeutic resistance in malignant cells and hasten defective cell removal [20, 21]. Iron metabolism dysregulation increases cancer risks and promotes tumor development. Iron addiction arises because cancer cells rely on iron more than normal cells [22]. Activating ferroptosis pathways may reverse drug resistance to current chemotherapy drugs, providing new treatment alternatives for cancer therapy. Ferroptosis produces metabolic dysfunctions that result in the generation of cytoplasmic and lipid ROS, which are not produced by mitochondria but, in certain cases, rely on NADPH oxidases [23]. Recent research created a metal-organic skeleton based on Fe^2+^ that delivers Fe^2+^ to cancer cells, causing Fenton reaction, excess ROS, and ferroptosis in BRCA cells [24]. Currently, the impact of lncRNA alterations on LUSC development remains elusive.

The present study obtained FRG expression knowledge and distinguished between mRNAs and lncRNAs. It was revealed that many lncRNAs were connected with FRGs in LUSC. 102 DEGs were found to be connected to ferroptosis. Research on the function of ferroptosis lncRNAs in LUSC found the prognostic validity of lncRNAs. C10orf55, AC016924.1, AL161431.1, LUCAT1, AC104248.1, and MIR3945HG were highly expressed in the high-risk group, suggesting their involvement in the oncology process of LUSC. Gu and Liu discover that high expression levels of AL161431.1 were observed in EC patients, tissues, and cells. Loss-of-function experiments validated the carcinogenic role of AL161431.1 [25]. Ma et al. found that lncRNA AL161431.1 was highly expressed in pancreatic cancer cells and tissues. Knockdown of lncRNA AL161431.1 led to increased cancer cell death and cell cycle arrest. Xenograft growth of SW1990 cells with stable knockdown of lncRNA AL161431.1 in mice was significantly slower than that of SW1990 cells with scrambled control shRNA [26]. Moreover, AP006545.2 and AL122125.1 were considerably higher in the low-risk group, implying the potential of these genes as LUSC tumor suppressor genes. Liu et al. identified AL122125.1 as a risk gene for LUSC by constructing an autophagy-related prediction model [27]. The biomarkers listed above may serve as therapeutic targets for LUSC. lncRNAs were also linked to patient outcomes in the LUSC trial. However, no definite proof was available to confirm their role in the synthesis of critical transcription factors linked with ferroptosis regulation [22, 28, 29].

The article "Identification of Clinical Prognostic Regulators and Analysis of Ferroptosis-Related Signatures in the Tumor Immune Microenvironment in Lung Squamous Cell Carcinoma" was retracted in 2023. Reasons: unreliable results or conclusions; lack of ethics approval or compliance; concerns about the data; concerns about the peer review.

The KEGG analysis demonstrated that the genes were predominantly engaged in ferroptosis, HIF-1, and the NOD-like receptor signaling pathway. Studies indicate that miRNAs and lncRNAs play essential roles in ferroptosis regulation. Nrf2 reduces the formation of reactive oxygen species via lowering iron absorption. miRNA prevents ferroptosis by controlling Nrf2 expression. In addition, miRNAs regulate iron transit, storage, utilization, and absorption [30–32]. Autophagy-dependent ferroptosis cancer cell death is regulated by the interaction of MTOR and GPX4 signaling [33]. HIF-1 is common in cancer-associated fibroblasts, and HIF-1-expressing fibroblasts activate the NF-B signaling pathway, increasing the growth of lung cancer tumors [34]. Zhang et al. [35] found that targeting CAFs that express HIF-1 might be a promising anticancer treatment.

Ferroptosis-related lncRNAs were strongly correlated with LUSC prognosis. Current research discovered eight lncRNAs related to prognosis and presented different expression levels in 2 at-risk people. Some lncRNAs were overexpressed in high-risk people (*p* < 0.05). Low-risk lncRNAs suggested superior results. Few studies on lncRNA changes linked to ferroptosis have been undertaken. Further research is necessitated to probe into the mechanism of ferroptosis-related lncRNA alteration, which will aid in the validation of our findings.

CCR, HLA, inflammation-promoting, parainflammation, T cell coinhibition, T cell costimulation, type I IFN response, and type II IFN response substantially infiltrated tumor tissues in the high-risk population. The findings may contribute substantially in a variety of therapeutic settings. lncRNAs appear to be effective markers for predicting LUSC patient outcomes. The relationship between lncRNAs and immune function was investigated. An association of several cell death mechanisms with anticancer immunity was found. In ICI-resistant tumors, the use of ICIs to induce ferroptosis and necroptosis led to increased anticancer effectiveness. The present study found the upregulation of checkpoint genes such as TMIGD2, TNFRSF4, CD244, NRP1, CD276, ICOS, and CD80, indicating their potential role as ICIs in LUSC. The connection of ICIs to ferroptosis receives little exploration. lncRNAs are linked to the control of these elements' expressions [36]. Based on the information presented above, it could be inferred that ferroptosis-related lncRNA alterations are related to LUSC progression.

The article "Identification of Clinical Prognostic Regulators and Analysis of Ferroptosis-Related Signatures in the Tumor Immune Microenvironment in Lung Squamous Cell Carcinoma" was retracted in 2023. Reasons: unreliable results or conclusions; lack of ethics approval or compliance; concerns about the data; concerns about the peer review.

NOD-like receptors have a role in inflammatory responses that aggravate the incidence and progression of respiratory organ transformation [37]. Based on the features outlined above, ferroptosis-related lncRNAs may control LUSC cell migration and proliferation via altering the NOD-like receptor signaling pathway. The low-risk population has better survival versus high-risk populations. The present approach anticipates LUSC patient survival with high accuracy. Risk score increases are associated with increased mortality and a higher high-risk ratio. The strategy in the present study had little impact on other indicators with possible implications for treatment outcomes. Ferroptosis-related lncRNAs appear to be useful biomarkers for therapeutic results prediction for LUSC.

The relationship between ferroptosis and LUSC has been marginally explored [38, 39]. Jie Yao et al. identified a 7-gene signature based on probable predictive ferroptosis regulatory genes, and these genes (ARHGEF26-AS1, LINC01137, C20orf197, MGC32805, TMPO-AS1, LINC00324, and LINC01116) were found to be negatively associated with LUAD clinical stage. The ferroptosis score is a promising biomarker that could be of great significance to determine the prognosis, molecular subtypes, TME cell infiltration characteristics, and immunotherapy effects in patients with LUAD by Weiju Zhang et al. The following is the study's novelty. First, the current study complemented prior papers with additional FRG data from the TCGA database, which is constantly updated. Second, to strengthen the credibility of the results, several databases were employed to measure immune cells and function. The current study has the following limitations: diverse data sources from other public resources were unavailable to validate the model's trustworthiness. Furthermore, only early expression investigation on the signature's 8 risk-lncRNAs was concentrated.

## 5. Conclusions

The findings contribute to the knowledge of the immune system's function in ferroptosis and lncRNA, perhaps providing an opportunity for novel effective therapies and predictive indications. The results may aid in the identification of lncRNAs that stimulate LUSC development, revealing their potential role in the process and advancement of LUSC carcinoma.

In addition, the purpose of this research is to identify and completely profile the gene signatures of ferroptosis-lncRNA-related regulators in LUSC. The several m6A alteration patterns greatly contributed to the TME's diversity and complexity. A prediction algorithm based on the m6a gene signature was also developed, which may predict the clinical course of LUSC. Our findings imply that the m6A genes are interesting prognostic indicators that might help guide effective immunotherapy and provide new insights into LUSC treatment choices.

The article "Identification of Clinical Prognostic Regulators and Analysis of Ferroptosis-Related Signatures in the Tumor Immune Microenvironment in Lung Squamous Cell Carcinoma" was retracted in 2023. Reasons: unreliable results or conclusions; lack of ethics approval or compliance; concerns about the data; concerns about the peer review.

## Figures and Tables

**Figure 1:** GO and KEGG analyses: (a) GO; (b) KEGG. 102 DEGs were identified (35 down- and 67 up-). GO analysis revealed 655 core targets.

**Figure 2:** Forest plot. There are 29 lncRNAs associated with the prognosis of LUSC; lncRNAs such as C10orf55 and AC016924.1 were freelance LUSC prognosis indices.

**Figure 3:** lncRNA signature. (a) Curve result. (b) AUC of risk factors. (c) DCA. (d) Risk survival status. (e) AUC of survival rate. (f) Heatmap.

**Figure 4:** COX analysis: (a) univariate, (b) multivariate, and (c) lncRNA and mRNA expression.

**Figure 5:** The heatmap for the prognosis signature. C10orf55, AC016924.1, AL161431.1, LUCAT1, AC104248.1, and MIR3945HG were found in the high-risk group. AP006545.2 and AL122125.1 were found in the low-risk group.

**Figure 6:** A hybrid nomogram. The hybrid nomogram was accurate, which demonstrated great potential in the therapy of LUSC patients.

**Figure 7:** GSEA analyses.

**Figure 8:** A heatmap for immune responses.

**Figure 9:** (a) Immune cell subpopulations. (b) Immune checkpoint.

**Figure 10:** The expression of FRGs in LUSC risk groups.

**Table 1:** The clinical characteristics of patients.

Variable	Number of samples
Sex	
Male/female	373/131
Age at diagnosis	
≤65/>65	190/314
Grade	
G1/G2/G3/G4/NA	Unknown
Stage	
I/II/III/IV/NA	245/163/85/7/4
T	
T1/T2/T3/T4	114/295/71/24
M	
M0/M1/NA	414/7/83
N	
N0/N1/N2/N3/NA	320/133/40/5/6

## Data Availability

No data were used to support this study.
